This article has been retracted.

# Digital inclusive finance, consumer consumption and high-quality economic development

**DOI:** 10.1371/journal.pone.0285695

**Published:** 2023-08-24

**Authors:** Wei Li, Hui Wang, Lu Zhang, Runchen Liu

**Affiliations:** 1 School of Accounting and Finance, Anhui Xinhua University, Anhui, China; 2 Taiwan Research Institute, Xiamen University, Xiamen, China; University of Galway, Ireland / Anhui University of Finance and Economics, CHINA

## Abstract

Against the backdrop of the COVID-19 pandemic and China’s pursuit of the "double circulation" strategy, scholars are increasingly focusing on ensuring high-quality economic development in China. In this regard, digital inclusive finance and consumer consumption are of utmost significance. This study employs panel data from 30 provinces and cities spanning 2011 to 2020 to explore the impact of digitized inclusive finance on consumer consumption and high-quality economic development through a spatial econometric model. Our findings indicate that integrating digital finance with consumer consumption and economic development fosters high-quality economic growth. Furthermore, our semi-parametric spatial lag model suggests a nonlinear relationship between digital inclusive finance and high-quality economic growth, shaped like an inverted "U". Additionally, we examine the mediating effect of consumer consumption on the relationship between digital inclusive finance and high-quality economic development. Our results reveal a substitution effect between digital inclusive financing and consumer consumption in promoting high-quality economic development. Therefore, it is essential to promote the development of digital inclusive finance, harness its positive spillover effects between regions, and encourage an increase in consumer consumption to optimize the consumption structure, upgrade and adjust the industrial structure, and spur growth in emerging industries.

## 1. Introduction

Since the initiation of China’s reform and opening-up policy, the country has experienced substantial economic growth and improvement in the living standards of its people. However, this progress has come at a cost, characterized by high pollution and energy consumption, leading to the emergence of serious environmental issues such as global warming. With the economy’s continuous development, Chinese people have raised their expectations for a higher quality of life, necessitating the exploration of approaches that promote high-quality economic development while prioritizing environmental protection.

The 19th National Congress of the Communist Party of China in 2017 acknowledged that the primary contradiction within Chinese society was unbalanced and inadequate development, along with the ever-growing needs of the people for an enhanced standard of living. The Congress proposed a shift in the economic development mode, emphasizing the need for swift high-quality economic growth. The concept of high-quality economic development encompasses diverse fields, necessitating coordinated efforts across all domains.

Scholars have extensively researched the primary challenges hindering high-quality development in China, which include uneven and insufficient economic growth. This challenge is manifested in the central and western regions of the country, which exhibit slower development than the eastern region, which has better resources and a thriving economy. To address this issue, inclusive finance has emerged as a viable solution aimed at providing effective financial services to marginalized groups such as small and micro-enterprises, low-income earners, and the poor.

In recent years, digital inclusive finance has gained prominence, driven by advancements in internet technology, promoting information dissemination, improving the coverage of inclusive finance, and facilitating poverty eradication efforts. Digital inclusive finance has the potential to identify relevant groups accurately, provide them with the necessary financial support, and ultimately promote harmonious social development and sustainable economic growth. Additionally, digital inclusive finance can contribute to the growth in household consumption, which is one of the three key drivers of economic development. Previous economic models in China were characterized by low- and medium-end consumption. However, with continued economic development, people have become increasingly interested in high-quality consumption. Consequently, household consumption has become a crucial engine of economic growth, with its continuous expansion facilitating development across all economic sectors, boosting related industries, and generating employment opportunities.

Furthermore, as household consumption continues to expand, it drives the optimization and upgrading of consumption structures. This upgrading process is marked by increasing demand for quality consumer goods and heightened attention to factors such as brand, culture, and service. These developments are important for the promotion of high-quality economic development in China.

This study aims to investigate the relationship between digital inclusive finance, consumer consumption, and high-quality economic development in China using a spatial econometric model with panel data from 30 provinces and cities. In addition to examining the linear relationships between these variables, a semi-parametric spatial lag model is employed to investigate potential non-linear relationships. This study also analyzes an analysis of the mediating and moderating effects of consumer consumption on the relationship between digital inclusive finance and high-quality economic development. Finally, to test the robustness of the results, the study also replaces the 0–1 weight matrix with an economical weight matrix. The findings of this study are expected to provide valuable insights into the impact of digital inclusive finance on consumer consumption and high-quality economic development contributing to the ongoing efforts to develop a high-quality economy in China.

This study contributes significantly to the existing literature in several ways. First, it examines the association between digital inclusive finance, household consumption, and high-quality economic development from both linear and nonlinear perspectives. The semi-parametric spatial lag model used in this study enables a more comprehensive analysis of the dynamic change process, adding to the credibility of this study. Second, this study focuses primarily on investigating the relationship between digital inclusive finance, household consumption, and high-quality economic development and endeavors to explore the paths of influence among these factors, offering guidance for future scholars interested in exploring these pathways. Finally, this study expands upon prior research by not only treating inclusive finance and consumption as explanatory variables, but also examining consumption as both an intermediary and moderating variable, providing a more nuanced understanding of the relationship among these three factors.

## 2. Theoretical analysis and research hypotheses

### 2.1 Digital inclusive finance and high-quality economic development

In 2005, inclusive finance was introduced to promote equal access to financial services for all customers. With the advancement of Internet technology, digital inclusive finance has emerged. While there is limited research on the impact of digital inclusive finance on high-quality economic development, some scholars have examined the relationship between digital finance, digital economy, and high-quality development. For instance, Xiong Wang (2022) found that digital inclusive finance can help small and medium-sized technology-based enterprises alleviate financing constraints [1], while Jianwei Li (2022) noted that it can effectively alleviate SME financing constraints, with private and family businesses benefiting in particular [2]. Other studies have investigated the role of inclusive finance in promoting economic growth through an analysis of the endogenous growth theory (Jun He, 2019) and the impact of the digital economy on high-quality economic development from various perspectives (Ren Baoping, 2022; Zhan Wenqing, 2022; YAN Tao, 2022; Liu Jiaqi, 2022; Ge Heping, 2021) [3–7]. Wu (2021) investigated the impact of the Internet on energy-saving efficiency and found that it can promote energy conservation and emission reduction through technological progress, human capital, openness, and energy structure [8]. Zhao (2022) showed that the digital economy can enhance the technological development and human capital of cities, with significant spillover effects across regions [9]. Li (2022) and Du (2022) demonstrated that digital finance can reduce environmental pollution by promoting industrial structure upgrading and rationalization, with marketization and government support playing important roles in this process [10, 11]. Han (2022) examined the link between finance and innovative development and found that financial development can attract human capital and promote innovation within and across regions [12]. These studies provide valuable insights into the complex relationship between digital technology and economic and social development, highlighting the multifaceted nature of this phenomenon and its potential to foster high-quality growth and sustainability. Based on these findings, it is evident that digital inclusive finance can promote enterprise innovation, meet the capital needs of enterprise survival and development, and optimize and adjust industrial structures, thereby improving economic development. This study recommends the following actions to enhance the impact of digital inclusive finance on high-quality economic development:

**Hypothesis 1:** the development of high-quality economies can be effectively promoted by digital inclusive finance.

### 2.2 Digital inclusive finance and consumer consumption

Goods and services are essential components of consumer consumption, and involve monetary or virtual expenditures to meet people’s basic needs for survival, development, and enjoyment. Researchers have studied the increasing consumption of consumersfrom the perspective of digital inclusive finance. Ang (2011) studied the impact of financial policy on private consumption in India and found that financial repression policies are linked to a reduction in private consumption fluctuations, while a more open financial system can help suppress it [13]. Grossman (2014) discovered that digital finance could reduce potential power consumption by providing convenience to consumers [14]. Cioacă (2020) demonstrated that internet technology can reduce income gaps and promote resident consumption when deeply integrated into society [15]. Based on spatial correlation and data from 265 Chinese prefecture-level cities from 2011 to 2018, Wang (2022) found that residents could effectively maximize their consumption potential with digital inclusive finance [16]. Compared with the western region, the eastern and central regions showed a more significant impact on driving consumption levels and the spatial spillover effect. Additionally, digital inclusive finance can drive an increase in consumer consumption in first and second-tier cities compared to third and fourth-tier cities. Based on China’s provincial data from 2011 to 2017, Jiang (2020) empirically found that digital inclusive finance improves consumer consumption levels and optimizes consumption structures by reducing the income gap between urban and rural areas and optimizing the industrial structure [17]. Yi (2018) observed that the inclusion of digital finance in promoting economic growth is stronger for rural, middle-income, and underdeveloped households, and is influenced by the education level and cognitive ability of the household head [18]. Li (2022) contended that digital inclusive finance, as a distinctive form of finance, is a vital driver in augmenting household consumption. Empirical evidence confirms that it has a substantial effect on boosting rural consumption [10]. From a climate change perspective and with reference to the historical temperature of cities, He (2022) found that digital financial inclusion can not only raise farmers’ consumption but also promote consumption upgrading to a certain extent. Moreover, digital financial inclusion can enhance the ability of individuals to withstand climate change [19]. Zhao (2022) asserts that with the advancement of mobile payments in China, digital inclusive finance can invigorate residents’ consumption and enhance the happiness of vulnerable groups [20]. Luo (2022) scrutinizes the association between digital financial inclusion and consumption inequality in China and demonstrates that digital financial inclusion can promote consumption among low-income individuals and diminish the income gap [21]. According to Cheng (2022), consumption has played an increasingly substantial role in propelling the economy since China entered a new era. Rural income and consumption are crucial components of high-quality economic development [22]. Therefore, the inclusion of digital finance and stable financial policies contributes to consumer consumption levels and consumption structures by increasing residents’ incomes and the spatial spillover effect. The following conclusions were drawn from the above analysis:

**Hypothesis 2:** Digital inclusive finance can effectively promote consumer consumption.

### 2.3 Digital inclusive finance, consumer consumption and high-quality economic development

China’s current economic development strategy is characterized by high-quality economic development, which not only focuses on the total amount of economic development but also develops an economic system that emphasizes quality. Scholars are studying innovative, coordinated, green, open, and shared developments to achieve this goal. Consumer consumption is considered an efficient means to achieve high-quality economic development through the use of digital inclusive financing. The Keynesian demand theory stresses that insufficient consumption demand will causes overcapacity and restrains economic growth. Rostow believed that only through consumption can industrial development and upgrading be stimulated to promote economic development at a more advanced level. Through theoretical analysis, Wang (2017) suggested through a theoretical analysis that China’s sustainable economic development needs to ensure economic growth through consumption, which is also an inevitable choice for future development in China [23]. Zhao (2020) found via model testing that China’s total consumption maintained a positive correlation with its economic growth and that the economic scale would continue to grow with the growth of total consumer consumption [24]. Through empirical analysis, Ma (2007) found that consumer consumption has a significant guiding and driving effect on China’s economic growth, and that the change in the consumer consumption structure will also force the upgrading and adjustment of the industrial structure [25]. Popescu (2010) and Lan(2022) argued that while the economy is important, maintaining a high quality of life requires healthy consumption patterns [26, 27]. Shu (2021) emphasized that the COVID-19 pandemic has significantly impacted China’s economy and highlighted the need to promote economic transformation, expand domestic demand, and achieve sustainable development driven by consumption [28]. Xing (2023) found that consumption upgrading can improve agricultural green total factor productivity and promote the long-term, high-quality development of alcoholometers through technical efficiency and progress [29]. Finally, Zhou (2022) contended that to cope with the pressure of sustainable economic development, it is crucial to improve consumption levels, and that digital payment methods can more effectively increase rural consumption and promote the upgrading of the consumption structure [30]. The existing research has confirmed that consumer consumption is crucial to economic growth. Additionally, the fusion of financial technology and financial development has improved range, precision, and efficiency leading to an increase in consumer income levels. In the context of "double-loop" development, China is increasingly demanding expanding domestic demand, breaking away from dependence on foreign trade, and promoting economic development. This study proposes a conclusion based on the above analyses.

**Hypothesis 3:** Consumer consumption mediates the relationship between digital inclusive finance and high-quality economic development.

A schematic illustrating the mechanism of digital inclusive finance, household consumption, and high-quality economic development is presented in Fig 1.

**Fig 1:** Mechanism analysis diagram.

In summary, the analysis of existing literature reveals two main gaps. Firstly, previous research has primarily focused on the relationship between digital inclusive finance, household consumption and high-quality economic development, with limited studies examining the linkages between the three variables, resulting in gaps in related research. Secondly, scholars in prior studies have not adequately considered the impact of digital inclusive finance on surrounding regions or the nonlinear relationship between the variables. Thus, this paper addresses these gaps by building upon previous studies and providing a more detailed examination of the relationship between digital inclusive finance, household consumption, and high-quality economic development. Consequently, this research makes a substantial contribution to the theoretical understanding and policy recommendations of the topic at hand.

## 3. Model setting and data description

### 3.1 Model construction

#### 3.1.1 Model setting based on spatial panel regression

China’s rapid economic growth, driven by reforms and opening-up, has been accompanied by unbalanced and uneven development among provinces, leading to a spatial clustering of high-quality economic development at the national level. In this study, we employ a spatial econometric model to investigate the effects of digital inclusive finance on consumer consumption and high-quality economic development, we employ a spatial econometric model in this study. Specifically, we use a spatial Durbin model based on the test results of the model, with the following specifications: (1)-(3):

$${\mathrm{CEE}}_{it}=\beta_{1}W_{i}{\mathrm{DIF}}_{it}+\beta_{2}{\mathrm{URE}}_{it}+\beta_{3}{\mathrm{GBE}}_{it}+\beta_{4}{\mathrm{CPI}}_{it}+\beta_{5}{\mathrm{EOI}}_{it}+\beta_{6}{\mathrm{CPE}}_{it}+u_{i}+\gamma_{i}+\varepsilon_{it}$$

$$\varepsilon_{it}=\lambda W_{i}\varepsilon_{t}+v_{it}$$ (1)

$${\mathrm{HQE}}_{it}=\beta_{1}W_{i}{\mathrm{DIF}}_{it}+\beta_{2}{\mathrm{URE}}_{it}+\beta_{3}{\mathrm{GBE}}_{it}+\beta_{4}{\mathrm{CPI}}_{it}+\beta_{5}{\mathrm{EOI}}_{it}+\beta_{6}{\mathrm{CPE}}_{it}+u_{i}+\gamma_{i}+\varepsilon_{it}$$

$$\varepsilon_{it}=\lambda W_{i}\varepsilon_{t}+v_{it}$$ (2)

$${\mathrm{HQE}}_{it}=\beta_{1}W_{i}{\mathrm{CEE}}_{it}+\beta_{2}W_{i}{\mathrm{DIF}}_{it}+\beta_{3}{\mathrm{URE}}_{it}++\beta_{4}{\mathrm{GBE}}_{it}+\beta_{5}{\mathrm{CPI}}_{it}+\beta_{6}{\mathrm{EOI}}_{it}+\beta_{7}{\mathrm{CPE}}_{it}+u_{i}+\gamma_{i}+\varepsilon_{it}$$

$$\varepsilon_{it}=\lambda W_{i}\varepsilon_{t}+v_{it}$$ (3)

Where *u*_*i*_ represents the individual effect, *γ*_*i*_ is the time effect, *λ* is the spatial autocorrelation coefficient, *β*_1_⋯*β*_7_ are the regression coefficients, *W*_*i*_ is the spatial weight matrix, *ε*_*it*_ and *v*_*it*_ is the error terms.

To better analyze the nonlinear relationship between digital inclusive finance, consumer consumption, and high-quality economic development, this paper proposes a semi-parametric spatial lag model with the following settings: (4)—(5):

$${\mathrm{CEE}}_{it}=\delta \sum_{j\neq i}W_{ij}{\mathrm{CEE}}_{it}+g({\mathrm{DIF}}_{\mathrm{it}})+\beta_{1}{\mathrm{URE}}_{it}+\beta_{2}{\mathrm{GBE}}_{it}+\beta_{3}{\mathrm{CPI}}_{it}+\beta_{4}{\mathrm{EOI}}_{it}+\beta_{5}{\mathrm{CPE}}_{it}+u_{i}+\gamma_{i}+\varepsilon_{it}$$ (4)

$${\mathrm{HQE}}_{it}=\delta \sum_{j\neq i}W_{ij}{\mathrm{HQE}}_{it}+g({\mathrm{DIF}}_{\mathrm{it}})+\beta_{1}{\mathrm{URE}}_{it}+\beta_{2}{\mathrm{GBE}}_{it}+\beta_{3}{\mathrm{CPI}}_{it}+\beta_{4}{\mathrm{EOI}}_{it}+\beta_{5}{\mathrm{CPE}}_{it}+u_{i}+\gamma_{i}+\varepsilon_{it}$$ (5)

Where *δ* is the spatial lag utility coefficient, and *g*(DIF_it_) is the non-parametric part. By taking the partial derivative of this formula, the nonlinear relationship between the development of digital inclusive finance on consumer consumption and high-quality economic development is obtained.

#### 3.1.2 Model setting based on mediating effect and moderating effect

It is essential to consider the mediating role of consumer consumption in the relationship between digital inclusive financing and high-quality economic development This study uses a mediating effect model to determine whether consumer consumption influences economic quality development. The specific models are shown in Eqs (6)–(8). Additionally, to evaluate whether the role of consumer consumption interferes with the relationship between digital inclusive finance and economic quality development, a moderating effect model was constructed as follows:

$${\mathrm{CEE}}_{it}=\beta_{1}{\mathrm{DIF}}_{it}+\beta_{2}{\mathrm{URE}}_{it}+\beta_{3}{\mathrm{GBE}}_{it}+\beta_{4}{\mathrm{CPI}}_{it}+\beta_{5}{\mathrm{EOI}}_{it}+\beta_{6}{\mathrm{CPE}}_{it}+u_{i}+\gamma_{i}+\varepsilon_{it}$$ (6)

$${\mathrm{HQE}}_{it}=\beta_{1}{\mathrm{DIF}}_{it}+\beta_{2}{\mathrm{URE}}_{it}+\beta_{3}{\mathrm{GBE}}_{it}+\beta_{4}{\mathrm{CPI}}_{it}+\beta_{5}{\mathrm{EOI}}_{it}+\beta_{6}{\mathrm{CPE}}_{it}+u_{i}+\gamma_{i}+\varepsilon_{it}$$ (7)

$${\mathrm{HQE}}_{it}=\beta_{1}{\mathrm{CEE}}_{it}+\beta_{2}{\mathrm{DIF}}_{it}+\beta_{3}{\mathrm{URE}}_{it}+\beta_{4}{\mathrm{GBE}}_{it}+\beta_{5}{\mathrm{CPI}}_{it}+\beta_{6}{\mathrm{EOI}}_{it}+\beta_{7}{\mathrm{CPE}}_{it}+u_{i}+\gamma_{i}+\varepsilon_{it}$$ (8)

$${\mathrm{HQE}}_{it}=\beta_{1}{\mathrm{CEE}}_{it}+\beta_{2}{\mathrm{DIF}}_{it}+\beta_{3}{\mathrm{CEE}}_{it}*{\mathrm{DIF}}_{it}+\beta_{4}{\mathrm{GBE}}_{it}+\beta_{5}{\mathrm{CPI}}_{it}+\beta_{6}{\mathrm{EOI}}_{it}+\beta_{7}{\mathrm{CPE}}_{it}+u_{i}+\gamma_{i}+\varepsilon_{it}$$ (9)

### 3.2 Variable selection

#### 3.2.1 Measurement of the level of high-quality economic development

Indicators of high-quality economic development should reflect many aspects, such as the continuous improvement of people’s lives and the steady development of the country’s economy. This study adopts the methods proposed by Zhang (2022), Shen (2022), and Wei (2022) to select 35 basic indicators to measure the level of high-quality economic development [31–33]. The specific indicators are listed in Table 1, which presents an indicator system for high-quality economic development.

**Table 1:** Indicator system of high-quality economic development.

Dimensions	Sub-index	Basic indicators	Indicators to measure the	Attribute
Innovative development	Innovation input	Research and development investment level	R&D investment/regional GDP	positive
		Level of researcher input	Full-time equivalent of R&D personnel/number of employees employed	positive
	Innovation output	Number of patents granted per capita	Number of patents granted/number of resident population	positive
		Percentage of technology market turnover	Technology market turnover/R&D investment	positive
Harmonious development	Regional coordination	Regional income ratio	Per capita disposable income of provincial residents/per capita disposable income of national residents	positive
		Regional consumption ratio	Per capita annual consumption of provincial residents/per capita annual consumption of national residents	positive
	Urban-rural coordination	Regional income ratio	Ratio of per capita annual disposable income of urban and rural residents	negative
		Urban-rural consumption ratio	Ratio of per capita annual consumption of urban and rural residents	negative
		Urban and rural fixed asset investment ratio	Ratio of fixed asset investment of urban and rural residents	negative
	Industrial harmony	Advanced industrial structure	Output value of tertiary industry/output value of secondary industry	positive
	Investment and consumption coordination	Rate of investment	Fixed asset investment/regional GDP	positive
		Consumption rate	Consumption expenditure/regional GDP	positive
		Investment consumption ratio	Investment in fixed assets/consumption expenditure	positive
Green development	Green production	Energy consumption per unit of output	Standard coal consumption/regional GDP	negative
		Exhaust emissions per unit of industrial added value	Industrial waste gas emissions/total industrial output value	negative
		Discharge of wastewater per unit of industrial added value	Industrial wastewater discharge/total industrial output value	negative
		Waste discharge per unit of industrial added value	Industrial waste discharge/total industrial output value	negative
	Green living	Domestic rubbish disposal	Harmless disposal rate of household garbage	positive
		Number of nature reserves	Number of nature reserves	positive
		Area of nature reserve	Area of nature reserve	positive
		Forest area	Forest area	positive
		Forest coverage rate	Forest coverage rate	positive
		Spending on environmental protection	Spending on environmental protection	positive
Open development	Trade openness	Opening-up in investment	Total import and export volume/ regional GDP	positive
	Opening-up in investment	Proportion of foreign direct investment	Total actual utilized foreign capital/ regional GDP	positive
Shared development	Benefit sharing	Number of public libraries	Number of public libraries	positive
		Per capita expenditure on education	Education expenditure/number of students in school	positive
		Per capita financial expenditure on medical and health care	Medical and health expenditure/ resident population	positive
		Number of doctors per 10,000 people	Number of doctors per 10,000 people	positive
		Number of hospitals and health centers per 10,000 people	Number of hospitals and health centers per 10,000 people	positive
		Per capita social security expenditure	Social security expenditure/number of resident populations	positive
	Financial Shared	Financial depth	(Deposits from financial institutions + loans from financial institutions)/ regional GDP	positive
		Financial breadth	Value added of financial sector/ regional GDP	positive
		Insurance penetration	Premium income/regional GDP	positive
		Width of insurance	Premium income/national premium income	positive

#### 3.2.2 Variable description

We selected the digital inclusive finance development index and consumer consumption as explanatory variables. The degree of development and the balance of digital inclusive finance are used to reflect the level of development. Additionally, a high-quality economic development index was chosen as the explanatory variable. To ensure the accuracy of our empirical model, we included several control variables: the urbanization rate, the general budget expenditure, consumer price index, investment efficiency, and capital production efficiency. Table 2 summarizes a summary of the selected variables.

**Table 2:** Calculation of variables and data sources.

Variable name	Variable meaning	Construction method
HQE	High-quality economic development	The improved entropy weight method is used to measure the economic high-quality development index
CEE	Consumer consumption expenditure	Consumption level of urban and rural residents
DIF	Digital inclusive finance	From Peking University Digital Inclusive Financial Index
URE	Urbanization rate	Urban population/total population
GBE	General budget expenditure	Log of general budget expenditures
CPI	Consumer Price index	The relative logarithm of the price change trend and degree of consumer goods and service items purchased by urban and rural residents in a certain period
EOI	Investment efficiency	National income growth/capital investment for fixed asset fund and current production fund growth
CPE	Capital production efficiency	Net benefits/costs

The 14th Five-Year Plan and the Outline of the Long-term Goals for 2035 both emphasized the need to develop China’s urbanization to a higher level. This urbanization drive is expected to boost the building material market and promote economic growth. As a result, the level of urbanization can influence consumer consumption and high-quality economic development. Therefore, we included the urbanization rate as one of the control variables in this study.

General budget expenditure refers to the planned allocation and use of centralized budget revenue by the state. This covers various fields such as capital construction, science and technology development, support for rural areas, and cultural and educational undertakings.

This expenditure plays a significant role in promoting infrastructure construction, industrial upgrading, the integrated development of urban and rural areas, and other dimensions of high-quality economic development. Therefore, it was considered a significant control variable in this study.

The Consumer Price Index reflects the changes in the prices of goods and services that are related to residents’ daily lives. An increase in the CPI indicates rising prices, which can have a significant impact on residents’ daily lives and economic development if sustained over time.

Investment efficiency measures the benefits of capital construction investments from perspective of the national economy perspective. This can effectively avoid inefficient and ineffective allocation of production factors, resulting in a waste of resources. Therefore, improving investment efficiency is crucial for sustainable economic development.

Capital production efficiency can be effectively measured as the output generated per unit of capital over time. This indicates that as output steadily increases, the production efficiency of capital improves, resulting in enhanced economic and social development. This reflects an improvement in the quality of economic development over time.

## 4. Empirical analysis

### 4.1 Data selection and processing

The main focus of this study was on panel data from 30 provinces, autonomous regions, and municipalities in China, covering the period from 2011 to 2020. Data from Tibet, Hong Kong, Macao, and Taiwan were excluded. Any missing data were filled in using the trendupdating method. Table 3 summarizes the descriptive data.

**Table 3:** Descriptive statistics of the variables.

Variable	Obs.	Mean	Std. Dev.	Min	Max
DIF	300	2.267	0.290	1.263	2.635
CEE	300	4.255	0.182	3.869	4.762
HQE	300	0.374	0.059	0.213	0.550
URE	300	58.207	12.099	34.960	89.600
GBE	300	3.635	0.253	2.849	4.238
CPI	300	102.573	1.196	100.600	106.300
EOI	300	0.361	0.121	0.127	1.060
CPE	300	1.413	0.721	0.266	4.158

### 4.2 Measurement of high-quality economic development index

The improved entropy weight method was used to derive an index of high-quality economic development after calculating 35 specific indicators in five dimensions. The results of high-quality economic development indices for China’s provinces and cities are presented in Table 4 and Fig 2, respectively, which provide a comprehensive summary of the specific results.

**Fig 2:** The economic high-quality development index of China’s provinces and cities.

**Table 4:** High-quality economic development index.

Region	2011	2012–2015	2016	2017	2018	2019	2020
Beijing	0.484	......................	0.563	0.564	0.57	0.584	0.572
Tianjin	0.364	......................	0.514	0.506	0.509	0.513	0.505
Hebei	0.305	......................	0.451	0.455	0.468	0.477	0.466
Shanxi	0.265	......................	0.407	0.393	0.41	0.412	0.414
Inner Mongolia	0.3	......................	0.467	0.464	0.484	0.48	0.488
Liaoning	0.336	......................	0.458	0.445	0.464	0.462	0.461
Jilin	0.295	......................	0.457	0.455	0.48	0.486	0.467
Heilongjiang	0.323	......................	0.492	0.5	0.506	0.514	0.506
Shanghai	0.405	......................	0.518	0.529	0.516	0.511	0.499
Jiangsu	0.375	......................	0.504	0.507	0.509	0.516	0.515
Zhejiang	0.409	......................	0.53	0.532	0.541	0.548	0.542
Anhui	0.298	......................	0.445	0.45	0.454	0.47	0.464
Fujian	0.345	......................	0.497	0.5	0.501	0.509	0.501
Jiangxi	0.318	......................	0.466	0.468	0.475	0.483	0.474
Shandong	0.348	......................	0.473	0.473	0.484	0.488	0.485
Henan	0.318	......................	0.463	0.464	0.478	0.485	0.475
Hubei	0.308	......................	0.48	0.483	0.486	0.498	0.485
Hunan	0.314	......................	0.48	0.485	0.486	0.499	0.493
Guangdong	0.413	......................	0.54	0.559	0.581	0.607	0.58
Guangxi	0.29	......................	0.463	0.457	0.473	0.481	0.476
Hainan	0.298	......................	0.455	0.457	0.449	0.46	0.458
Chongqing	0.299	......................	0.468	0.468	0.462	0.472	0.475
Sichuan	0.342	......................	0.494	0.502	0.51	0.52	0.51
Guizhou	0.216	......................	0.408	0.417	0.421	0.436	0.424
Yunnan	0.278	......................	0.466	0.471	0.472	0.481	0.472
Shaanxi	0.292	......................	0.467	0.469	0.468	0.484	0.48
Gansu	0.224	......................	0.366	0.413	0.411	0.413	0.405
Qinghai	0.269	......................	0.451	0.464	0.453	0.428	0.439
Ningxia	0.214	......................	0.415	0.415	0.411	0.415	0.414
Xinjiang	0.263	.....................	0.33	0.34	0.347	0.353	0.358

Table 4 and Fig 1 illustrate the varying levels of high-quality economic development across China’s provinces and cities. As of 2020, Guangdong Province (0.579), Beijing (0.571), and Zhejiang Province (0.541) had the highest index values for high-quality economic development. In contrast, the three provinces and cities with the lowest index values were the Ningxia Hui Autonomous Region (0.413), Shaanxi Province (0.413), and Gansu Province (0.404). The level of high-quality economic development of different regions in China varies depending on their geographical location. The eastern region, located in a relatively superior geographic area, ranks first in terms of high-quality economic development. The central region has achieved steady economic growth rates and high-quality development levels in the eastern region. However, the western regions have relatively slow economic development owing to their geographical location and environment, resulting in a lower level of high-quality economic development than the eastern and central regions. Generally, the eastern regions exhibit a higher level of high-quality economic development than the western and central regions at the national level.

### 4.3 Spatial econometric regression results

#### 4.3.1 Spatial autocorrelation test

Prior to conducting the spatial econometric regression, it was necessary to examine the presence of spatial autocorrelation in the variables. Spatial autocorrelation is commonly assessed using the Moran’s index, which measures the degree of similarity between the values of a variable in adjacent regions. A Moran’s index greater than zero indicates a positive spatial correlation, whereas a negative value indicates a negative spatial correlation. As shown in Table 5, the Moran indices for high-quality economic development, digital inclusive finance, and consumer consumption were positive and statistically significant from 2011 to 2020, suggesting a strong spatial association between these variables in China’s provinces and cities. Therefore, this study employed spatial econometric techniques to explore these relationships.

**Table 5:** Global Moran index of high-quality economic development.

Year	High-quality economic development	Digital inclusive finance	Consumer consumption
2011	0.451*** (0.000)	0.438*** (3.856)	0.403*** (0.000)
2012	0.458*** (0.000)	0.449*** (4.009)	0.375*** (0.000)
2013	0.435*** (0.000)	0.433*** (3.878)	0.368*** (0.000)
2014	0.432*** (0.000)	0.431*** (3.869)	0.342*** (0.001)
2015	0.373*** (0.000)	0.368*** (3.353)	0.349*** (0.001)
2016	0.418*** (0.000)	0.427*** (3.85)	0.350*** (0.001)
2017	0.478*** (0.000)	0.491*** (4.393)	0.360*** (0.001)
2018	0.521*** (0.000)	0.537*** (4.738)	0.361*** (0.000)
2019	0.529*** (0.000)	0.545*** (4.789)	0.359*** (0.001)
2020	0.552*** (0.000)	0.569*** (4.983)	0.358*** (0.001)

Note: ***, **, * indicate significance at the levels of 1%, 5%, 10% respectively.

Based on the scatter plot of the Moran index in 2020 (Figs 3–5), it is evident that there was a spatial correlation between high-quality economic development, consumer consumption, and digital inclusive finance among provinces and cities in China during the epidemic period. This positive correlation can be attributed to the government’s scientific and reasonable epidemic prevention measures, which minimized the impact of the epidemic on the economy.

**Fig 3:** Scatter plot of Moran index of high-quality development in 2020.

**Fig 4:** Scatter plot of Moran index of consumer consumption in 2020.

**Fig 5:** Scatter plot of Moran index of digital inclusive finance in 2020.

### 4.4 Empirical results of spatial panel regression

In this study, the spatial weights were calculated using a 0–1 matrix, where a value of 1 indicates adjacency between two provinces and 0 indicates otherwise. To determine the appropriate spatial econometric model to use, we conducted a joint significance test as well as the LR and LM tests (Table 6). The p-value of R-LM (lag) was 0.343 when studying the impact of digital inclusive finance on quality economic development quality, and the other variables are significant. This suggests that the spatial error model can be inferred preliminarily. Subsequently, based on the results of both the LR and WALD tests, the spatial Durbin model was recommended as it is more general than spatial error or spatial lag models. Although the selected models of the LM, LR, and LM tests were not consistent, the spatial Durbin model was recommended. Therefore, we recommend using the spatial Durbin model with time and double-fixed variables after conducting Hausman and joint significance tests.

**Table 6:** Test results of spatial econometric model.

statistic	Model (1)		Model (2)		Model (3)	
	statistic	P values	statistic	P values	statistic	P values
Moran’s I	3.402***	0.001	3.268***	0.001	3.356***	0.001
LM (error)	164.467***	0.000	150.360***	0.000	153.466***	0.000
R-LM (error)	164.112***	0.000	146.686***	0.000	149.959***	0.000
LM (lag)	0.765	0.382	4.574**	0.032	4.285**	0.038
R-LM (lag)	0.409	0.522	0.900	0.343	0.778	0.378
Wald_lag	66.080***	0.000	40.760***	0.000	47.770***	0.0000
Wald_error	64.540***	0.000	41.270***	0.000	47.950***	0.0000
LR_lag	59.880***	0.000	38.270***	0.000	44.440***	0.000
LR_error	17.940***	0.0030	38.340***	0.000	44.030***	0.000
Hausman	28.940***	0.0067	27.030**	0.0123	20.590	0.1503
Joint significance test (ind)	97.500***	0.000	67.490***	0.000	/	/
Joint significance test (time)	545.470***	0.000	626.290***	0.000	/	/

When examining the impact of digital inclusive finance on consumer consumption, the LM (lag) and R-LM (lag) p-values were 0.382 and 0.522, respectively. However, both the LR and WALD tests were significant, suggesting the use of the spatial Durbin model. As the selected models of the LM, LR, and LR tests were not consistent, the spatial Durbin model was recommended. This is because it is more general than the spatial error and spatial lag models. After conducting the Hausman and joint significance tests, we found that the spatial Durbin model with time and individual double fixation should be used.

When examining the impact of digital inclusive finance and consumer consumption on high-quality economic development, the p-value of R-LM (lag) was 0.378, and the remaining variables were significant. Subsequently, the LR and WALD tests found that both are significant, so spatial Durbin model can be used. Based on the Hausman test results, there was no significance found in the p-value of 0.150, and therefore, the random effects model was used to carry out the research.

When examining the impact of digital inclusive finance on high-quality economic development (as shown in Table 7), a positive correlation was found between digital inclusive finance and high-quality economic development. Specifically, an increase of 1% in digital inclusive finance resulted in a 4.3% increase in high-quality economic development, verifying Hypothesis H1. Additionally, an increase of 1% in the general budget for the control variables resulted in a 5.6% increase in high-quality economic development, suggesting a positive correlation between economic development and the general budget, with a higher budget level leading to better economic development. The reason for this may be that the shift in government spending from the general public budget to public investment, scientific and technological innovation, and environmental protection in China has prompted the improvement of infrastructure, increase of income, and enhancement of social welfare. As an important tool for adjusting income distribution, general public expenditure also contributes to the adjustment of the tax system and the reduction of the individual burden. This may explain why China has been able to achieve the goal of high-quality economic development, as general public expenditure plays a significant role in this process. When studying the impact of digital inclusive finance on consumer consumption, it was found that consumer consumption increased by 6.9% when digital inclusive finance increased by 1%, indicating a positive correlation between digital inclusive finance and consumer consumption. A higher level of digital inclusive finance leads to higher consumer consumption and vice versa, thus verifying H2. Among the control variables, investment efficiency was positively correlated with consumer consumption. Specifically, a 1% increase in investment efficiency will resulted in a 2.5% increase in consumer consumption. This may be due to the fact that an increase in investment efficiency raises the overall wealth level of society, increasing income expectations and boosting consumption. Meanwhile, the level of general budget expenditure was negatively correlated with consumer consumption, with a 1% increase in general budget expenditure resulting in a 2.3% decrease in consumer consumption. This is due to effective investment efficiency as firstly, improvement in investment efficiency can directly contribute to economic growth and enhance people’s income and wealth levels but also inevitably influence the consumption level and consumption structure. Secondly, a high level of investment efficiency can help stabilize the economy, enhance market confidence, and encourage investors to spend freely. When examining how digital inclusive finance and consumer consumption contribute to high-quality economic development, it was found that a 1% increase in digital inclusive finance will results in a 3.066% increase in high-quality economic development and a 1% increase in consumer consumption leads to an 8.161% increase in high-quality economic development, which is significant at the 1% level. Therefore, digital inclusive finance and consumer consumption are positively related to high-quality economic development, with a stronger driving effect on high-quality economic development. Furthermore, the lower the level of digital inclusive finance and consumer consumption, the weaker the impact on high-quality economic development. Among the control variables, investment efficiency is negatively correlated with the consumer price index, possibly due to the increased efficiency of investment in certain manufacturing industries, the replacement of manual labor with more intelligent manufacturing equipment, and a decrease in expected income from wages. Additionally, the rise in the consumer price index affects consumer spending to some extent.

**Table 7:** Results of spatial Durbin regression.

Variable	Model (1)	Model (2)	Model (3)
CEE			0.082***(3.130)
DIF	2.550** (0.069)	0.043*** (3.260)	2.060** (0.031)
URE	0.003*** (3.800)	0.001 (1.320)	0.001* (1.790)
GBE	-0.023 (-0.590)	0.056*** (2.970)	0.094*** (7.240)
CPI	0.001 (0.280)	-0.001 (-0.780)	-0.001 (-0.220)
EOI	0.025 (1.160)	-0.001 (-0.100)	-0.015* (-1.310)
CPE	-0.006 (-1.220)	0.001 (0.500)	0.004 (1.780)
R^2^	0.925	0.745	0.923

Table 8 shows the model’s three spatial spillover effects, revealing a direct effect of 0.069 for digital inclusive finance on high-quality economic development, with a total effect of 0.109, but no significant indirect utility. This indicates that digital inclusive finance promotes economic development directly by impacting high quality, but not through regional spillover effects. According to Model (2), the direct effect of digital inclusive finance on consumer consumption was 0.044 and the total effect was 0.071, with no significant indirect utility. This suggests that digital inclusive finance enhances consumer consumption through a direct effect, but not through regional spillover effects. Based on the results of Model (3), it can be seen that the direct effect of digital inclusive finance on high-quality economic development was 0.030 and the total effect was 0.036, with no significant indirect effect. Additionally, the direct effect of consumer consumption on high-quality economic development was 0.083 and the total effect was 0.095, both of which were statistically significant at the 5% level. However, the indirect effect was not significant, indicating that the direct effect of consumer consumption on high-quality economic development was insignificant at the 5% level.

**Table 8:** Decomposition of spatial spillover effects.

	Model (1)			Model (2)			Model (3)		
variable	Direct effect	The indirect effect	The total effect	Direct effect	The indirect effect	The total effect	Direct effect	The indirect effect	The total effect
CEE							0.083*** (3.160)	0.011 (0.260)	0.094** (1.970)
DIF	0.069** (2.440)	0.041 (1.020)	0.109*** (3.240)	0.044*** (3.240)	0.028 (1.350)	0.071*** (3.850)	0.030** (2.210)	0.005 (0.330)	0.036*** (3.270)
URE	0.003*** (3.820)	-0.003 * (-1.860)	0.001 (0.420)	0.001 (1.320)	0.001** (1.990)	0.002** (3.050)	0.001** (2.210)	0.002 * (1.870)	0.002*** (2.970)
GBE	-0.024 (-0.650)	0.240*** (3.860)	0.215*** (3.390)	0.058*** (3.140)	-0.152*** (-4.620)	-0.094*** (-2.630)	0.090*** (7.150)	-0.073*** (-2.750)	0.017 (0.550)
CPI	0.001 (0.230)	0.005 (1.110)	0.005 (1.250)	-0.001 (-0.830)	-0.004* (-1.700)	-0.005** (-2.060)	-0.001 (-0.250)	-0.001 (-0.240)	-0.001 (-0.490)
EOI	0.025 (1.200)	-0.025 (-0.570)	0.001 (0.010)	0.001 (0.090)	0.022 (0.990)	0.021 (0.820)	-0.015 (-1.370)	-0.027 (-0.980)	-0.043 (-1.370)
CPE	-0.005 (-0.990)	-0.045*** (-4.070)	-0.050*** (-4.090)	0.001 (0.550)	0.012** (2.160)	-0.011* (-1.690)	0.004* (1.670)	-0.001 (-0.150)	0.003 (0.460)

### 4.5 Semi-parametric spatial lag model

The nonlinear relationship between digital inclusive finance and consumer consumption is shown in Fig 6 as an inverted U-shaped curve. The curve shows that When the level of digital inclusive finance development is below 2.4, it promotes positive consumer consumption. However, when high-quality economic development falls between the range of 2.4–2.6, the influence of digital inclusive finance on consumer consumption becomes weakens. On the one hand, digital inclusive finance provides consumers with more efficient and convenient financial services, enabling them to access more financial support, thereby promoting economic and consumption growth. On the other hand, the expansion of digital financial inclusion may lead to inappropriate marketing strategies and risky loans by financial institutions, resulting in a higher debt ratio for consumers, which can negatively affect their consumption levels. Nevertheless, the overall impact of digital inclusive financing on consumer consumption remains positive and mostly.

**Fig 6:** Partial map of digital inclusive finance on consumer consumption.

Fig 7 shows a nonlinear relationship between digital inclusive finance and high-quality economic development, characterized by an inverted U pattern. The figure illustrates that digital financial inclusion has a positive effect on economic quality development until it reaches a level of 2.3, beyond which digital financial inclusion begins to have a negative impact on economic quality development. In the initial stage of economic development, income augmentation through consumption can boost economic growth and drive the upgrade of the consumption structure. However, as consumer demand saturates, certain consumption patterns may have negative societal impacts, such as excessive borrowing and overconsumption. These behaviors can lead to financial distress, financial crises, and other problems that can be detrimental to sustainable economic growth. Overall, the influence of digital inclusion on high-quality economic development appears to gradually diminish and ultimately becomes negative beyond a certain threshold.

**Fig 7:** Partial map of digital inclusive finance on high-quality economic development.

### 4.6 Mediating effect

This study examined the mediating effect of consumer consumption on the relationship between digital inclusive finance and the quality of economic development. We conducted a secondary test using bootstrap statistics to ensure robustness of the results. As shown in Table 9, all the regression results were significant at the 5% level. However, relying solely on ordinary regression alone could lead to biased conclusions. Therefore, we also considered the spatial spillover effects between regions to make the regression results more descriptive. We used bootstrapping to test for the presence of a mediating effect, which was indicated if the 95% confidence interval did not include 0. Our results showed that there is a mediating effect, as neither the direct nor indirect effects included zero in the bootstrap tests. Thus, our results support H3, indicating that digital inclusive finance influences the quality of economic development through the mediating effect of consumer consumption.

**Table 9:** Mediating effect test results.

Variable	Model (6)	Model (7)	Model (8)
CEE			0.255*** (21.590)
DIF	0.397*** (13.920)	0.128*** (13.920)	0.027** (3.610)
_cons	3.355*** (52.140)	0.084*** (4.020)	-0.771*** (-18.480)
[95%Conf.Interval] (_bs_1)	(0.085, 0.117)		
[95%Conf.Interval] (_bs_2)	(0.012, 0.041)		
R^2^	0.394	0.400	0.764
Proportion of mediating effect	0.791		

This study introduces digital inclusive finance as an interaction term with consumer consumption to test the moderating effect, while considering the mediating effect. As shown in Table 10, the negative coefficient of the interaction term and the significantly positive coefficient of consumer consumption suggest that consumer consumption weakens the positive contribution of digital inclusive finance to high-quality economic development. The positive contribution of digital inclusive finance is more significant when consumer consumption is low. As the level of consumer consumption increases, the positive contribution of digital inclusive finance decreases. These findings indicate that consumer consumption has a significant substitution effect on the positive contribution of digital inclusive finance to high-quality economic development

**Table 10:** Results of moderating effect test.

Variable	Model (9)
CEE	0.193** (2.620)
DIF	0.200** (2.200)
DIF* CEE	-0.041* (-1.790)
URE	0.001 (0.540)
GBE	0.101*** (3.910)
CPI	0.001 (0.380)
EOI	-0.017 (-1.460)
CPE	0.005 (1.440)
_cons	-0.931* (-2.600)
R^2^	0.922

### 4.7 Robustness test

To ensure the robustness of our findings, we conducted a robustness test by using a geographical distance matrix instead of a 0–1 matrix for the weight matrix. Table 11 summarizes the results, which demonstrated that digital inclusive finance has a significant positive effect on high-quality economic development at the 1% significance level and a positive effect on consumer consumption at the 10% significance level. Significantly, the numerical values were consistent with those obtained from the to 0–1 matrix, suggesting that our spatial econometric analysis is robust.

**Table 11:** Spatial econometric results based on the geographical distance weight matrix.

Variable	Model (1)	Model (2)	Model (3)
CEE			0.065*** (2.6)
DIF	0.312*** (34.58)	0.021* (1.69)	0.024* (1.66)
URE	0.004*** (4.37)	0.001 (0.13)	2.05** (0.001)
GBE	0.006 (0.14)	0.058*** (3.17)	0.096*** (6.76)
CPI	0.0026 (0.83)	-0.001 (0.91)	-0.001 (-0.69)
EOI	0.037* (1.7)	0.006 (0.65)	-0.013* * (-1.22)
CPE	-0.006 (-1.2)	0.003 (1.32)	0.005 (2.28)
R^2^	0.898	0.741	0.923

As shown in Figs 8 and 9, when comparing the bias diagram of digital inclusive finance and the bias diagram of digital inclusive finance on high-quality economic development by changing the spatial weight matrix and using the 0–1 matrix, it can be found that the two bias diagrams are essentially the same. This indicates that the empirical results are not affected by changing the spatial weight matrix in the semi-parametric lag model, and thus the spatial lag model used in this paper is robust.

**Fig 8:** Partial map of geographic weight matrix digital inclusive finance on consumer consumption.

**Fig 9:** Partial map of geographical weight matrix digital inclusive finance on high-quality economic development.

## 5. Research conclusions and suggestions

The study aimed to investigate the correlation between digital inclusive finance, consumer consumption, and quality economic development in 30 provinces and cities in China from 2011 to 2020. The results suggest that: (1) There is a nonlinear relationship between digital inclusive finance and high-quality economic development, forming an inverted "U" shape. (2) Digital inclusive finance has a significant positive effect on public consumption, and the relationship between digital inclusive finance and public consumption also follows a nonlinear inverted "U" shape. (3) Consumer consumption mediate the relationship exists between digital inclusive finance and high-quality economic development. However, there is a significant substitution relationship between consumer consumption and digital inclusive finance in the development of a high-quality economy. Based on these findings, the following recommendations are proposed.

First, the regional network infrastructure should be improved to ensure the accessibility of digital financial inclusion products for a broader population. Second, financial literacy and knowledge should be popularized to increase overall financial participation by strengthening financial education and encouraging diversified product usage to gain value from capital break-even. Moreover, optimizing the environment for the development of digital inclusive finance is critical, including formulating relevant policies, standardizing market orders, and establishing a credit system to ensure sustainable and healthy development. Only through the implementation of these measures can we realize the positive spillover effects of digital financial inclusion on the economy and society.

Consumption is a crucial driver of economic growth, and plays an essential role in national development. Residents’ consumption demand is a significant source of economic growth. Improving the distribution system, strengthening the social security system, increasing residents’ income levels, and enhancing their purchasing power are necessary to promote consumption upgrades and growth. Moreover, the government can support consumer consumption by implementing preferential policies and other means of stimulating economic growth. Furthermore, optimizing the consumption structure can promote the upgrading and optimization of industrial structures. The structure and patterns of household consumption can directly affect an enterprise’s production and supply. Therefore, guiding consumers to adopt sustainable and green products and services can promote industrial upgradation, reduce environmental pollution and resource waste, and increase society’s overall well-being. Additionally, consumption increases residents’ sense of happiness and fulfillment, thereby promoting social harmony and stability. Thus, the government should strengthen consumer protection, maintain market order, crack down on illegal acts that infringe on consumers’ rights and interests, enhance their confidence, and protect their rights and interests to play a positive role in social harmony and stability. The government should also formulate corresponding policies to strengthen consumption-oriented industrial policies and support and encourage the development of green industries, such as environmental protection, energy conservation, low carbon, and new energy. This will guide consumers towards a sustainable and low-carbon lifestyle and enhance social awareness and a sense of responsibility for environmental protection.

This study examined the relationships between digital inclusive finance, household consumption, and high-quality economic development. However, it has several limitations: (1) Although the paper highlights the connection between digital inclusive finance, household consumption, and high-quality economic development, there may be additional transmission paths among the three. Moreover, there may not be a simple one-way causal relationship between variables but a more intricate two-way causal relationship. Therefore, a more precise definition of the relationship between these two is required. (2) Indicators of high-quality economic development must be explicit. As China has recently proposed high-quality economic development, it has not yet formed a completely unified index system; therefore, the indicators should be more accurate. Given these concerns, future research will include more theoretical logic on the relationship between digital inclusive finance, resident consumption, and high-quality economic development. The Granger causality test was used to determine the causal relationships between them. Finally, as China develops, a high-quality economic development indicator system can be defined more accurately, allowing the establishment of a more precise indicator system.

## Supporting information

S1 Data (XLSX)
